# An exploratory study of structural and microvascular changes in the skin following electrical shaving using optical coherence topography

**DOI:** 10.1111/srt.13830

**Published:** 2024-07-01

**Authors:** Pakhi Chaturvedi, Wilco Kroon, Giulia Zanelli, Peter R. Worsley

**Affiliations:** ^1^ Skin Sensing Research Group School of Health Sciences, University of Southampton Southampton UK; ^2^ Philips Consumer Lifestyle B.V. Drachten The Netherlands

**Keywords:** cheek, electrical shaving, forearm, neck, optical coherence tomography, sensitive skin

## Abstract

**Background:**

Consumer products such as electrical shavers exert a combination of dynamic loading in the form of pressure and shear on the skin. This mechanical stimulus can lead to discomfort and skin tissue responses characterised as “Skin Sensitivity”. To minimise discomfort following shaving, there is a need to establish specific stimulus‐response relationships using advanced tools such as optical coherence tomography (OCT).

**Objective:**

To explore the spatial and temporal changes in skin morphology and microvascular function following an electrical shaving stimulus.

**Methods:**

Ten healthy male volunteers were recruited. The study included a 60‐s electrical shaving stimulus on the forearm, cheek and neck. Skin parameters were recorded at baseline, 20 min post stimulus and 24 h post stimulus. Structural and dynamic skin parameters were estimated using OCT, while transepidermal water loss (TEWL) was recorded to provide reference values for skin barrier function.

**Results:**

At baseline, six of the eight parameters revealed statistically significant differences between the forearm and the facial sites, while only surface roughness (Rq) and reflectivity were statistically different (*p* < 0.05) between the cheek and neck. At 20 min post shaving, there was a significant increase in the TEWL values accompanied by increased blood perfusion, with varying magnitude of change dependent on the anatomical site. Recovery characteristics were observed 24 h post stimulus with most parameters returning to basal values, highlighting the transient influence of the stimulus.

**Conclusions:**

OCT parameters revealed spatial and temporal differences in the skin tissue response to electrical shaving. This approach could inform shaver design and prevent skin sensitivity.

## 1 INTRODUCTION

More than 50% of the population regard themselves as individuals with sensitive skin.^1^ This could be attributed to greater recognition/evidence of symptoms or even increased interest in cosmetics and the general maintenance of healthy skin.^2^ As such, there is an escalation in the demand for personalised products and interventions to promote skin health.^3^ Sensitive skin continues to be an active area of interest in both industry and medicine/dermatology research fields, with direct application to cosmetic product design and medical interfaces.^4^

With respect to mechanical stimulation of the skin, consumer products such as electrical shavers interact with the skin while exerting a combination of dynamic loading in the form of pressure, friction and shear. When subjected to an external force, the skin as a whole can be considered a viscoelastic material with different mechanical properties in lateral and vertical directions that depend on the loading conditions and indentation depth.^5^ It has long been established that in certain users, shaving can cause redness, inflammation, acne and other symptoms associated with skin sensitivity.^6^ Pseudo‐folliculitis barbae (PFB) is a common inflammatory reaction of the hair follicle, most often on the neck region resulting from shaving. Also known as ‘razor bumps' or ‘shaving bumps', it can also occur on any site where hair is shaved or plucked, including the axilla, pubic area and legs. This often manifests in acne‐like symptoms presenting as ingrown hairs associated with flesh‐coloured or red follicular papules. However, research to date on the prevalence and impact of these skin reactions has been limited to predominantly questionnaire‐based evaluation on consumer panels.^7^ To meet the demands for personalised products and interventions to promote skin health, there is a need to establish individual thresholds of tolerance to external mechanical stimuli and work towards personalised solutions to promote skin health. By incorporating scientific measurement and imaging technology, insights could be gained into both the perceived and observed aetiology of shaving sensitivity and skin symptoms.^4^

Optical coherence tomography (OCT) has been identified as a potential tool for assessing a range of structural and physiological skin parameters.^4^ Its combination of image resolution and depth of penetration makes it suitable for dermatological applications.^8^, ^9^, ^10^, ^11^, ^12^, ^13^ Indeed, researchers have developed algorithms to digitally analyse OCT images, extracting details such as skin layer thickness and surface roughness (Rq).^13^, ^14^, ^15^, ^16^, ^17^, ^18^ In recent years OCT has been used to characterise morphological and physiological changes in skin aging. The results from an observational study included a significantly decreased dermal attenuation coefficient and trends of increased roughness with age.^19^ The authors concluded that the technology has the potential to personalize therapies based on objective findings. Indeed, in a recent systematic review and meta‐analysis OCT was shown to improve the detection of persistent basal cell carcinoma (BCC) after medical treatment.^20^ Despite its reported potential, there are limited studies exploring the application of OCT in mechanical skin damage and subsequent recovery.

One of the recent advances which could expand our understanding of temporal changes in skin physiology is dynamic optical coherence tomography (D‐OCT), which allows visualization of the skin vasculature by detection of motion from speckle variance.^21^ This non‐invasive imaging tool is able to visualize the epidermis, upper dermis and its blood vessels and evaluate epidermal thickness (ET) and blood flow. Studies have shown seasonal effects on blood vessel depth.^22^ and identified its potential to assess features of chronic wound healing.^23^ Thus, there is a strong potential to identify spatial and temporal changes in skin blood flow following the mechanical insult of shaving.

There is a paucity of published evidence regarding the structural and physiological changes in the skin following shaving, despite a high prevalence of skin sensitivity in specific anatomical locations, for example, the neck. Accordingly, the current study aimed to explore the spatial and temporal changes in skin morphology and microvascular function following an electrical shaving insult using a D‐OCT protocol.

## 2 METHODS

Healthy male volunteers were recruited from the local university population to participate in this exploratory repeated‐measure study. The study was approved by the local Faculty Ethics Committee of the University of Southampton (FoHS‐Ethics‐71825). The test protocol was performed in the Biomechanics Testing Laboratory in the Clinical Academic Facility at Southampton General Hospital, Southampton, UK. The room temperature was maintained at 22°C ± 2°C.

### 2.1 Test equipment and skin parameters

Transepidermal water loss (TEWL) was recorded to provide reference values for changes in skin barrier function as many studies have reported higher TEWL values following mechanical insults.^24^, ^25^, ^26^ An open chamber Tewameter (TM300, Courage and Khazaka, Germany) was used, which has been shown to have good reliability.^27^ and is accurate when compared to gold standard gravimetric testing.^28^ TEWL was measured by placing the device in gentle contact with the skin, where the value is determined from the average of the readings after a period of equilibrium was achieved. The final parameter was determined by the average of two repeated measurements, reported in grams per meter squared per hour (g/m^2^/h).

A Vivosight Dx system (Michelson Diagnostics, UK) was used for recording OCT scans of the skin. This is a multi‐beam Swept‐Source Frequency Domain OCT system that operates at an A‐line rate of 20 kHz. It has a 1300 nm centre wavelength, 7.5 µm lateral and 5 µm axial resolution. The image size is 1342 × 460 pixels captured at 20 frames per second. The OCT scan volume recorded was 4 × 4 × 2 mm^3^. Two repeated scans were conducted at each measurement point, with optimal spacing and minimal pressure applied to the skin surface during image capture.

The images obtained were subsequently analysed in the proprietary VivoTools software to determine morphological and dynamic skin parameters, namely, surface reflectivity ratio (SRR), plexus depth, vessel diameter and vessel density at 0.3 mm depth, highlighted in Figure 1A. D‐OCT also known as angiographic OCT, is based on the principles of speckle variance OCT. It visualizes the microvasculature in the superficial dermis.^13^, ^24^, ^26^ and may answer the demand for a non‐invasive, real‐time imaging method for local skin pathology.^21^, ^23^, ^29^, ^30^ Furthermore, the images were exported to MATLAB for estimation of the RMS variation of surface height (Rq). Additionally, A‐scans were derived for the 3D OCT stacks and the optical coefficient of the skin tissue was estimated using a previously reported algorithm.^31^ The corresponding Scaled Intensity Drop (SID) was estimated from the A‐scans where the peak intensity value (corresponding to the air‐skin interface) was normalized for the 3D stack. As highlighted in Figure 1B, the SID is defined as the coefficient of the slope of the signal between the skin surface to the point where the signal is reduced by 80%. In addition, A‐scans were analysed to estimate the Area under the Curve (AuC) up to 0.2 mm skin depth to quantify OCT signal attenuation of the superficial skin layers, as highlighted in Figure 1C.

**FIGURE 1:** Overview of skin parameters included in the present study as shown in the (A) annotated dynamic OCT image from the Vivosight OCT system; (B) and (C) A‐lines for the OCT scans extracted via MATLAB. Skin parameters include: 1. Plexus depth (µm), 2. Vessel diameter (µm), 3. Vessel density (%), 4. Surface reflectivity ratio, 5. RMS variation of surface height, Rq (µm), 6. Scaled Intensity Drop, SID (mm^−1^), 7. Area under the Curve, AuC (dB.mm). OCT, optical coherence tomography.

### 2.2 Mechanical stimulus

A shaving stimulus was given on the forearm, cheek and neck to investigate different anatomical sites. Following institutional ethical regulations, the shaver head was specifically modified for this project to provide a relatively high coefficient of friction to the skin of participants. Furthermore, a commercially available Philips shaving handle from the S9000 series was used in the study. The S9000 shaving handle was equipped with load sensors to estimate the amount of force applied onto the shaver head, which has been calibrated into colour options providing graded light feedback to the user for an optimal shaving experience. The participants were requested to shave for 60 s at each anatomical location and to apply the shaving contact pressure such that the light ring on the shaver handle was in the orange zone (corresponding to a high shaving pressure).

### 2.3 Measurement protocol

Participants were requested to clean shave 72 h before the test session using their normal shaving routine. Using a stencil (70 mm × 50 mm) with a cut‐out (15 mm × 15 mm), non‐permanent squares were drawn on the forearm, cheek and neck for each participant to standardize the location of measurement across multiple visits (Figure 2A). In particular, the hirsute regions of the cheek and neck were selected for this study. Skin parameters were recorded at baseline (BL), 20 min post stimulus (S + 0.3h) and 24 h post stimulus (S + 24h) to characterise recovery (Figure 2B).

**FIGURE 2:** (A) Region of interest highlighted on the forearms, cheek and neck; (B) Timepoints of the data collection: BL à Baseline; S + 0.3h à 20 min post stimulus; S + 24hr à 24 h post stimulus.

### 2.4 Statistical analysis

Data from each measurement device were exported to Excel and Minitab for visualization and statistics. Most parameters have a non‐significant Anderson–Darling normality test, indicating that the data were non‐normally distributed. Thus, non‐parametric statistics were used. Temporal responses on each anatomical site were analysed for differences from baseline using the Wilcoxon signed‐rank test. Furthermore, final recovery characteristics were also tested for statistical significance using the same statistics. Correlations between the skin parameters were investigated using the Spearman's correlation test. A 95% confidence interval was calculated for the OCT parameters.

## 3 RESULTS

Ten male volunteers were recruited for this study, as detailed in Table 1. The cohort was predominantly younger adults with ages ranging from 24 to 41 years. Results for TEWL values for P2 have not been included due to malfunctioning of the probe.

**TABLE 1:** Participant demographics including age and Fitzpatrick skin type.

Participant no.	Age (years)	Fitzpatrick skin type
P1	35	4
P2	28	3
P3	25	2
P4	37	5
P5	24	3
P6	38	3
P7	36	4
P8	37	3
P9	41	4
P10	41	3

### 3.1 Baseline comparison between skin sites

The median and quartile values for each baseline skin parameter are detailed in Table 2. Comparing the results from the forearm with those from the facial sites, six of the eight parameters revealed statistically significant differences (*p* < 0.05), namely TEWL, AuC, SRR, plexus depth, vessel diameter and vessel density. In addition, there were differences in the inter‐subject variability in these parameters. For example, vessel density on the facial sites revealed a much wider range of values (9.3%–18.5%) compared to the forearm (2.8%–4.9%). Interestingly, largely overlapping values between the cheek and neck skin were noted for the TEWL and dynamic vascular OCT parameters, demonstrating some equivalence of these facial sites at baseline. However, statistically significant differences between the cheek and neck were observed for three of the four structural OCT parameters, namely SID, Rq and SRR. For example, the median roughness at the neck was approximately 1.5 times greater than that at the other sites.

**TABLE 2:** Median, first quartile and third quartile values for all baseline skin parameters at each anatomical site at baseline.

	Forearm	Cheek	Neck
**Functional parameters**			
TEWL (g/m^2^h)	7.54^*^, ^***^ (6.66–10.61)	12.38^*^ (10.40–15.49)	11.32^***^ (11.00–14.64)
**Structural parameters**			
SID (mm^−1^)	1.53^*^ (1.40–1.56)	1.81^*^, ^**^ (1.70–1.95)	1.56^**^ (1.50–1.63)
AuC (a.u.)	13,824^*^, ^***^ (13,576–14,006)	12,602^*^ (11,935–13,366)	13,004^***^ (12,610–13,409)
Rq (µm)	13.3^***^ (12.1–14.9)	12.2^**^, ^***^ (9.0–13.9)	21.4^**^ (19.4–23.0)
SRR (a.u.)	1.06^*^, ^***^ (1.05–1.10)	1.17^*^, ^**^ (1.12–1.23)	1.03^**^, ^***^ (0.99–1.04)
**Dynamic parameters**			
Plexus depth (µm)	355^*^, ^***^ (345–372)	258^*^ (249–281)	279^***^ (240–313)
Vessel diameter (µm)	45^*^, ^***^ (35–52)	66^*^ (47–76)	62^***^ (55–85)
Vessel density (%)	3.3^*^, ^***^ (2.8–4.9)	14.3^*^ (11.3–18.5)	11.1^***^ (9.3–18.2)

*Note*: Statistically significant differences between anatomical sites were investigated using the Wilcoxon test (*p* < 0.05).

Abbreviations: AuC, Area under the Curve; Rq, surface roughness; SID, Scaled Intensity Drop; SRR, surface reflectivity ratio; TEWL, Transepidermal water loss.

* *p* < 0.05 between forearm and cheek.

** p < 0.05 between cheek and neck.

*** p < 0.05 between forearm and neck.

### 3.2 Temporal trends in skin barrier function following electrical shaving

In the present study, the skin's barrier functional response has been measured using TEWL (Figure 3A). It was observed that the shaving stimulus resulted in a significant increase in values on the cheek (median ∆TEWL = 3.3 g/m^2^h) and neck (median ∆TEWL = 34.5 g/m^2^h), with the former having a high inter‐subject variability (*p* < 0.05). Indeed, the neck skin demonstrated a 2.8 times increase from baseline in the post stimulus values, with results at S + 0.3h ranging from 12.7 to 91.9 g/m^2^h. Furthermore, recovery characteristics were also observed on the cheek and neck as the TEWL returned near basal values (results ranging from 9.36  to 19.66 g/m^2^h), revealing a significant decrease from S + 0.3h values (*p* < 0.05). However, P10 was observed as an outlier at S + 24h with TEWL equal to 36.89 g/m^2^h. In contrast, the forearm skin revealed no significant change in response to the stimulus such that results ranged from 5.65  to 15.19 g/m^2^h over each timepoint (*p* > 0.05).

**FIGURE 3:** Temporal response for functional parameters of the skin following shaving on the forearm cheek, and neck. Wilcoxon signed‐rank test (^*^ *p* < 0.05, ^**^ *p* < 0.01).

### 3.3 Temporal trends in the structural skin parameters

For the structural OCT parameters, the results for SID (Figure 3B) revealed statistically significant increases from baseline in post stimulus values on all anatomical sites (*p* < 0.05 on arm and cheek, *p* < 0.01 on neck). These differences represented site‐specific changes post‐stimulus (S + 0.3h), where SID ranged from 1.40  to 1.81 mm^−1^ on the forearm, 1.56  to 2.24 mm^−1^ on the cheek and 1.61  to 1.78 mm^−1^ on the neck. Furthermore, statistically significant recovery was observed only on the cheek and neck (*p *< 0.01).

In contrast, the AuC (Figure 3C) revealed differing statistical trends on each anatomical site. The forearm revealed no change following shaving and recovery (*p* > 0.05). Similarly, the cheek demonstrated small changes in values post stimulus. However, following the recovery period, AuC on the cheek was statistically greater than baseline and post stimulus values (median ∆ AuC = 340 a.u. and 747 a.u., respectively; *p* < 0.05). In contrast, the neck demonstrated a statistically significant decrease in AuC from baseline to S + 0.3h and recovery back to basal values from S + 0.3h to S + 24h (median ∆ AuC = 1203 a.u. and 1415 a.u., respectively; *p* < 0.01).

For Rq (Figure 3D), only the forearm revealed a decrease from baseline (median Rq = 13.25 µm) in values following shaving, such that the median post stimulus Rq = 11.5 µm (*p* < 0.01) and median recovery Rq = 10.4 µm (*p* < 0.05). In contrast, the cheek and neck demonstrated no significant changes in response to the stimulus. For SRR (Figure 3E), the forearm and neck revealed a statistically significant increase from baseline in post stimulus values such that the median ∆SRR was equal to 0.08 a.u. and 0.12 a.u., respectively (*p* < 0.05). Notably, there was a large inter‐subject variation in results on the neck at S + 0.3h as values ranged from 1.02 . to 1.21 a.u. Although recovery was observed on both sites, the results did not achieve significance (*p* > 0.05). In contrast, the cheek demonstrated no changes throughout the test period.

### 3.4 Temporal trends in the dynamic microvascular skin parameters

The vascular skin response to electrical shaving measured using D‐OCT was characterised using plexus depth, vessel diameter and vessel density. Results for the plexus depth (Figure 3F) revealed a prolonged influence of shaving on the forearm where values at S + 0.3h and S + 24h were significantly lower than those at baseline (median ∆ plexus depth = 14 µm, *p* < 0.05). By contrast, short‐term changes were observed on the neck associated with a decrease in plexus depth following stimulus (median ∆ plexus depth = 62 µm, *p* < 0.01), proceeded by a recovery (median ∆ plexus depth = 43 µm, *p* < 0.01). However, no significant changes were observed for the plexus depth on the cheek. It is of note that with respect to the vessel diameter (Figure 3G), the shaving stimulus revealed a significant increase in values only at the cheek site such that the median ∆ vessel diameter = 7 µm, *p* < 0.05. Vessel density (Figure 3H) revealed statistically significant increases from baseline in post stimulus values on each anatomical site. However, the relative change from baseline varied at each site such that the median ∆ vessel density was 1.3% on the forearm (*p* < 0.05), 4.9% on the cheek (*p* < 0.05) and 25.1% on the neck (*p* < 0.01). After 24 h, the values on the forearm remained elevated (*p* < 0.05 from baseline), while those on the neck revealed a statistically significant decrease (*p* < 0.01 from S + 0.3h).

### 3.5 Associations between skin parameters

There were significant correlations between the functional, structural and dynamic parameters when collated across all time points of investigation (Table 3). Notably, TEWL revealed moderate correlations with specific structural and dynamic OCT parameters highlighting its functional nature. For example, TEWL demonstrated a negative correlation with AuC (*r* = −0.519, *p* < 0.01) and plexus depth (*r* = −0.578, *p* < 0.01). In addition, most structural and dynamic parameters revealed significant correlations within their respective sub‐groups. Interestingly, SRR demonstrated statistically significant correlations with six of the seven other parameters, although its association with dynamic parameters was weak.

**TABLE 3:** Summary of the Spearman's rank correlation coefficients between measurement parameters.

	Functional parameter	Structural parameter				Dynamic parameter	
	TEWL (*n* = 52)	SID (*n* = 58)	AuC (*n* = 58)	Rq (*n* = 58)	SRR (*n* = 58)	Plexus depth (*n* = 58)	Vessel diameter (*n* = 58)
**Structural parameters**							
SID	*r* = 0.213 *p* = 0.13						
AuC	*r* = −0.519 *p* < 0.01	*r* = −0.398 *p* < 0.01					
Rq	*r* = 0.151 *p* = 0.28	*r* = −0.805 *p* < 0.01	*r* = 0.097 *p* = 0.47				
SRR	*r* = 0.337 *p* = 0.02	*r* = 0.553 *p* < 0.01	*r* = −0.556 *p* < 0.01	*r* = −0.543 *p* < 0.1			
**Dynamic parameters**							
Plexus Depth	*r* = −0.578 *p* < 0.01	*r* = −0.362 *p* = 0.01	*r* = 0.688 *p* < 0.01	*r* = 0.041 *p* = 0.76	*r* = −0.255 *p* = 0.05		
Vessel Diameter	*r* = 0.061 *p* = 0.67	*r* = −0.14 *p* = 0.29	*r* = 0.148 *p* = 0.27	*r* = 0.073 *p* = 0.59	*r* = −0.268 *p* = 0.04	*r* = −0.086 *p* = 0.52	
Vessel Density	*r* = 0.648 *p* < 0.01	*r* = 0.107 *p* = 0.43	*r* = −0.408 *p* = 0.24	*r* = 0.157 *p* = 0.24	*r* = 0.111 *p* = 0.41	*r* = −0.705 *p* < 0.1	*r* = 0.411 *p* < 0.01

*Note*: Pairs with *p* < 0.05 have been highlighted in bold with shades of light to dark blue for ascending positive *r* values and shades of light to dark red for descending negative *r* values.

Abbreviations: AuC, Area under the Curve; Rq, surface roughness; SID, Scaled Intensity Drop; SRR, surface reflectivity ratio; TEWL, Transepidermal water loss.

## 4 DISCUSSION

With respect to the development of consumer products designed to interact with the skin, there is a need to establish an objective relationship between stimuli and local tissue response. The aim of the current study was to explore the spatial and temporal changes in skin structure and function following an electrical shaving stimulus. The authors note that the shaving device used for the mechanical stimulation was a prototype specifically developed for this project that provided a high coefficient of friction at the skin/device interface. D‐OCT imaging was employed to characterise morphological and physiological skin responses, giving a unique perspective on skin changes following complex mechanical loading. The observations revealed a significant variation at baseline between anatomical sites and distinct changes across many of the parameters immediately following shaving. The recovery characteristics also differed between sites, with the most notable changes in the skin barrier, skin morphology and microvascular properties observed on the neck site. This corroborates common self‐reported signs of shaving dermatitis and PFB.^32^

Distinct anatomical sites were investigated, evaluating the spatial variability in skin response to shaving. At baseline, the magnitude of values for the vessel diameter and vessel density were smaller on the forearm than on the cheek/neck. Conversely, the plexus depth on the forearm was greater when compared to the cheek/neck, indicating that the vasculature on the facial sites is more superficial and denser than the forearm. The surface topography data showed the lowest roughness values on the forearm, similar to other studies.^13^ These results indicate that the forearm skin may not be a suitable proxy for the cheek/neck skin when investigating the influence of mechanical stimuli pertinent to shaving. Furthermore, the anatomical sites of primary interest in this research included the bearded skin on the cheek and neck for males. The results offer novel data, creating opportunities for future studies examining characteristics of hirsute skin, especially as there is a paucity of studies reporting values for facial skin of healthy males.^33^ Thus, this data are considered crucial for the development of skin‐contacting devices as results from broader studies examining differences in skin parameters with reference to gender, race and anatomical sites have reported conflicting results.^34^, ^35^, ^36^, ^37^, ^38^, ^39^, ^40^, ^41^

With respect to the structural skin parameters, site and time dependent changes were observed, showing the local effects of shaving stimulus. Of note, the data revealed that the neck skin was significantly rougher than the cheek and forearm skin at baseline, while the shaving stimulus resulted in significant changes in roughness for up to 24 h only on the forearm. To the best of our knowledge, we are the first to report these differences following a shaving stimulus between the cheek and neck skin. From our data, the cheek revealed higher SID and SRR values than the neck following shaving. As the attenuation of the OCT signal is influenced by the presence of micro vessels and structural elements such as collagen fibres,^42^ the results indicate that the neck had a denser dermis which may have been combined with a less strong signal from the stratum corneum (SC). However, as the SRR estimates the relative intensity of the top surface of the skin to that of the dermis, a denser dermis is expected to yield lower SRR values. As such, it is unclear whether the SC or the dermis properties are driving the SRR change.

Several baseline parameters demonstrated largely overlapping values between the cheek and neck skin, demonstrating some equivalence of these facial sites. However, differences were observed in the skin response to shaving. For example, the dynamic skin parameters such as plexus depth revealed significant changes due to shaving only on the neck skin. It has been hypothesised that shaving‐induced skin irritation is most likely a result of mechanically induced neurogenic inflammation with reflex hyperaemia, which may be caused by microtrauma.^32^ Our study corroborates this hypothesis with distinct changes in microvascular parameters measured using dynamic OCT. However, further research is needed to elicit its relationship to inflammatory markers, which could include the use of non‐invasive biofluids from the skin surface.^43^ No direct comparative studies were found in the literature to corroborate this finding. One study.^44^ examined the basal blood flow in skin tissue on several facial sites using laser Doppler flowmetry and, similar to the presented results, did not reveal any statistically significant differences between the cheek and neck. Another study.^45^ investigated the changes in blood flow on the finger following tape stripping using optical microangiography (OMAG), revealing significantly increased blood flow at 1 min post stimulus which recovered after 15 min.^30^ The results found in this study suggest that there is a distinct hyperaemic response in the local tissues following mechanical stimulus, where superficial tissue becomes perfused via microvascular recruitment as part of a physiological reaction. This could be associated with local damage to the epidermal and dermal tissues, where blood can transport platelets and leukocytes to facilitate coordinated and cooperative activities in normal healing that limit acute inflammation and trigger tissue repair.^46^ However, additional research investigating the vasculature of facial skin is needed to understand the differences in the skin response to mechanical stimuli such as shaving.

The present study also examined correlations between the various parameters, confirming the common use of TEWL as a suitable indicator of the functional status of the skin. Indeed, it is widely reported that mechanical stimulation in the form of tape stripping results in an increase in TEWL, corresponding to a compromise of the functional integrity of the SC.^47^, ^48^, ^49^ However, as the functional difference between the skin on the cheek and neck remains unclear, the anatomical variations in the TEWL response in the present study implicate the interaction of the stimulus with the skin surface. It is possible that the density and direction of beard hair varied between the two sites leading to differences in the subsequent skin tissue response. Reportedly, the neck skin is rougher than the cheek and the hair has a lower emerging angle.^32^ These factors may contribute to the stimulus introduced in the present study where participants were requested to shave in a small area for 60 s There may also be differences in the pre‐conditioning of these skin sites, with cheek skin exposed to environmental challenges (UV, wind, rain) more frequently than the neck site. This may alter the tolerance to external stimuli.

## 5 LIMITATIONS

Analysis of the results was not generalisable due to a small cohort size of 10 participants. Future research should include a diverse population of participants from a wide age range, which has been shown to influence the structure and function of facial skin using OCT parameters.^19^ It is noted, that the present study used SID to characterise the optical properties of the skin, rather than the VivoTools generated parameter, Optical Attenuation Coefficient (OAC).^19^, ^50^ Statistical equivalence was established between the two and SID was selected for further investigation allowing comparative analysis with internal studies. On the contrary, AuC analysis was developed due to limitations in VivoTools, where it failed to detect the thickness of the epidermis in a majority of the dataset. Upon closer inspection, it was noted that the A‐scans did not have a clear peak at the dermal‐epidermal junction (DEJ). Similar features were observed by other researchers, which has been attributed to the digital smoothing of the wavy DEJ as the A‐lines are averaged.^42^ Additionally, the presented results only examined structural and dynamic parameters of the skin. In the context of enhanced skin sensitivity and the development of skin‐friendly consumer products, the authors believe it is crucial to consider biophysical, biochemical and perceived changes in the skin tissue to build a holistic model of skin response to specified stimuli.

## 6 CONCLUSION

The authors believe that the present study is unique in using D‐OCT to investigate the response of the hirsute skin of the cheek and neck in response to electrical shaving. The shaving insult resulted in a decrease in the barrier function (as measured by TEWL) accompanied by increased blood perfusion, with the magnitude of these responses differed between anatomical sites, most notably the greatest change was observed at the neck. Furthermore, recovery characteristics were observed 24 h post stimulus as most parameters returned to basal values, highlighting the transient influence of such mechanical stimuli. As such, these findings can be further investigated towards developing site‐specific skin‐friendly devices.

## Data Availability

The data that support the findings of this study are openly available in Dataset A consumer study to evaluate the skin's response at https://eprints.soton.ac.uk/481027/, reference number https://doi.org/10.5258/SOTON/D2743.
